The article "The Relationship between Urinary Stones and Gut Microbiomeby 16S Sequencing" was retracted in 2024. Reasons: signs of a paper mill; suspected computer-generated content; unreliable results or conclusions; concerns about the data.

# The Relationship between Urinary Stones and Gut Microbiomeby 16S Sequencing

**DOI:** 10.1155/2020/1582187

**Published:** 2020-10-05

**Authors:** Chenhao Zhou, Kai Li, Lun Zhao, Wei Li, Zongbao Guo, Jingyao Xu, Xiaofei Qi, Hexing Yuan

**Affiliations:** Department of Urology Surgery, The First Affiliated Hospital of Soochow University, Soochow, China

## Abstract

**Objective:**

To understand the relationship between urinary stones and the gut microbiome and to screen for microbial species that may be involved in stone formation.

**Methods:**

Stool samples were collected from patients with urolithiasis and healthy patients between March and December 2017. The samples were analyzed by 16S sequencing to determine differences in the microbiome profiles between the two groups. The mouse model was established and was divided into two groups. Fecal samples were collected from the mice before gavage and three weeks postgavage for microbiome analysis. The microbial population of each group was analyzed to screen for microbial species that may affect the formation of urinary stones. Differences in the number of crystals in the renal tubules of the mice were examined by necropsy.

**Results:**

The microbial composition was different between urolithiasis patients and healthy controls. The urolithiasis patients had significantly reduced microbial abundance; however, increased proportions of Bacteroidetes and Actinobacteria were detected compared to healthy controls. Furthermore, the abundance of Alistipesindistinctus and Odoribactersplanchnicus was significantly increased in the urolithiasis patients compared to the healthy controls. In addition, the incidence of urolithiasis was much higher in the experimental mouse group (stone solution + urolithiasis patient stool) than in the control mouse group. However, the microbial abundance before gavage was not significantly different from that seen three weeks postgavage.

**Conclusion:**

Theurolithiasis patients in this study had a different gut microbiome when compared with that of healthy individuals. The altered microbiome increased the rate of crystal formation in renal tubules and accelerated urinary stone formation in the mouse model of urolithiasis.

## 1. Introduction

Urolithiasis is a common disease among inpatients in the division of urology. Epidemiological studies from Europe and the U.S. have shown that 5%-10% of individuals develop urinary stones at least once in their lifetime. In recent years, the incidence of urolithiasis has been increasing in China and the country now has one of the three highest incidences of urolithiasis in the world. As our understanding of the etiology of urolithiasis deepens, metabolic risk factors for urinary stones have gained increased attention from urologists.

The article "The Relationship between Urinary Stones and Gut Microbiomeby 16S Sequencing" was retracted in 2024. Reasons: signs of a paper mill; suspected computer-generated content; unreliable results or conclusions; concerns about the data.

The scientific community has demonstrated great interest in the study of the gut microbiome in recent years. Studies have shown that the gut microbiome is associated with numerous human diseases but its role in the pathophysiology of urolithiasis is not known. A recent study found that the composition of the gut microbiome was significantly different between urolithiasis patients and nonurolithiasis patients [1]. However, it is unclear whether the difference in microbial abundance between urolithiasis patients and controls was the cause of stone formation or the consequence of other factors, such as antibiotic exposure and diet [2]. In 1985, Allison et al. reported that Oxalobacterium formigenes (Oxf) was involved in the formation of calcium oxalate stones [3]. However, the potential impact of other microbial species on urolithiasis has been rarely investigated. Therefore, this study is aimed at examining the effect of the gut microbiome and its mechanism of action in urinary stone formation in order to provide a basis for further research in this area.

## 2. Materials and Methods

### 2.1. Materials

#### 2.1.1. Experimental Animals

Twenty clean grade healthy adult mice were purchased from Shanghai SLAC Laboratory Animal Co., Ltd. Experimental animal welfare and ethics review were conducted, and the study was approved by the Animal Ethics Committee of Soochow University.

#### 2.1.2. Reagents and Instrument

An Olympus optical microscope was used in this study. Ethylene glycol and ammonium chloride were obtained from Sigma-Aldrich.

#### 2.1.3. Preparation of Main Solutions

*(1) Urolithiasis-Inducing Solution (Stone Solution)*. 5 ml ethylene glycol and 5 g ammonium chloride were dissolved in 500 ml phosphate-buffered saline (PBS).

*(2) Stone Solution + Urolithiasis Patient Stool*. Stool samples were collected from urolithiasis patients and homogenized in distilled water. After particulates in the solution settled, the supernatant was collected and mixed with the stone solution.

*(3) Stone Solution + Healthy Control Stool*. Stool samples were collected from patients in the Division of Urology without a history of urolithiasis and homogenized in distilled water. After the particulates in the solution settled, the supernatant was collected and mixed with the stone solution.

*(4) Stone Solution + Mouse Feces*. Mouse feces were homogenized in equal volumes of distilled water. After particulates in the solution settled, the supernatant was collected and mixed with stone solution. This solution was used as a control.

*(5) Stone Solution + PBS*. PBS and an equal volume of supernatant were mixed with stone solution.

*(6) Urolithiasis Patient Stool Solution*. Stool samples were collected from urolithiasis patients and homogenized in distilled water. After particulates in the solution settled, the supernatant was collected and numbered to identify them.

*(7) Healthy Control Stool Solution*. Stool samples were collected from patients in the Division of Urology without a history of urolithiasis and homogenized in distilled water. After particulates in the solution settled, the supernatant was collected and numbered to identify them.

*(8) Mouse Fecal Solution*. Mouse feces were homogenized in an equal volume of distilled water. After particulates in the solution settled, the supernatant was collected and numbered.

The article "The Relationship between Urinary Stones and Gut Microbiomeby 16S Sequencing" was retracted in 2024. Reasons: signs of a paper mill; suspected computer-generated content; unreliable results or conclusions; concerns about the data.

### 2.2. Methods

### 2.3. Sample Collection

Stool samples were collected from patients diagnosed with urolithiasis in our hospital between March and December 2017 (experimental group) and from patients without urolithiasis treated in the Division of Urology during the same period (control group). Five patients from the experimental group were paired with five patients in the control group, and the urolithiasis and non-urolithiasis patient pairs were gender-matched and within two years of age. The selected patients in the experimental group were test10, test15, test43, test56, and test63. The selected patients in the control group were control_5, control_6, control_7, control_11, and control_12.The fecal microbiomes of the patients were analyzed by 16S sequencing.

Twenty healthy adult mice were randomly divided into four groups of five mice per group. The mice in each group were fed different solutions ((1) stone solution + urolithiasis patient stool, (2) stone solution + mouse feces, (3) stone solution + healthy control stool, and (4) stone solution + PBS) for four weeks. The mice were euthanized by cervical dislocation, placed in a supine position, and the abdomen was sterilized with 75% alcohol. The skin and muscle layers were incised using surgical scissors and forceps to expose the organs. The abdominal fat was gently pulled toward the head of the mouse by forceps to expose the kidneys, which were then harvested, fixed in 10% formalin, and numbered.

#### 2.3.1. Diagnostic Criteria for Urolithiasis

Patients who met any one of the following diagnostic criteria was definitively diagnosed with urolithiasis: (1) patients with stone shadows by X-ray, (2) the indication of stones by ultrasound, or (3) surgical removal of stones or excretion of stones from the urethra following extracorporeal lithotripsy. Exclusion criteria include kidney failure, urinary tract malformations, urinary tract infections, and hyperthyroidism.

The article "The Relationship between Urinary Stones and Gut Microbiomeby 16S Sequencing" was retracted in 2024. Reasons: signs of a paper mill; suspected computer-generated content; unreliable results or conclusions; concerns about the data.

#### 2.3.2. Inclusion Criteria for the Control Group

Patients in the Division of Urology who were previously healthy were included in the control group.

#### 2.3.3. Exclusion criteria

Patients with a history of systemic disease, urinary stones, or other urinary tract diseases were excluded from the control group.

### 2.4. Statistical Analysis

All data were statistically analyzed using SPSS software (SPSS Inc., Chicago, IL, United States). Counted data are expressed as the number of cases or percentage and were compared between groups using the *χ*^2^ test. *P* < 0.05 was considered statistically significant.

## 3. Results

### 3.1. Differences in the Microbiome

The Shannon index curves of the microbial profiles of the 10 experimental and control group patients are shown in Figure 1.

As shown in Figure 1, the Shannon index distribution was significantly different among the experimental and control groups, except for control 6; control 6 was a patient with an open fracture. The patient underwent surgery and received antibiotics upon admission, and the stool sample was collected after surgery. Therefore, the deviation in this patient may be attributable to the effect of antibiotics on the gut microbiome.

The proportions of Bacteroidetes and Firmicutes were significantly different between the healthy controls and urolithiasis patients (Figure 2).

#### 3.1.1. Effect of the Microbiome on Stone Formation

Mice were fed four different stone solution mixtures for four weeks. Upon euthanization by cervical dislocation, the spleens were collected and examined. The number of renal tubules containing crystals and the ratio of crystal-containing tubules to the total number of tubules were calculated and compared among the samples.

As shown in Figure 3, mice fed stone solution + urolithiasis patient stool had significantly higher crystal-containing tubule to total tubule ratios than the other three groups. In addition, the crystal-containing tubule to total tubule ratio varied among all four groups, indicating that the urolithiasis patient stools accelerated the rate of crystal formation and hence stone formation in the renal tubules of mice.

#### 3.1.2. Analysis of Microbial Species

We identified 400 microbial species belonging to the Bacteroides, Heliobacillus, Clostridium, and Fusobacterium genera.

Figures 4 and 5 show differences in the Shannon index and phylum between the eight groups. Group 2 (urolithiasis patient stool) and group 6 (mouse feces after urolithiasis patient stool gavage) had significantly higher Shannon indices than the other groups. At the phylum level, group 2 (urolithiasis patient stool) had significantly increased proportions of Proteobacteria and Fusobacteria than group 1 (healthy control stool), a difference also seen between group 5 (mouse feces before urolithiasis patient stool gavage) and group 6 (mouse feces after urolithiasis patient stool gavage). These findings further support our earlier conclusion.

The article "The Relationship between Urinary Stones and Gut Microbiomeby 16S Sequencing" was retracted in 2024. Reasons: signs of a paper mill; suspected computer-generated content; unreliable results or conclusions; concerns about the data.

#### 3.1.3. Screening of Target Species

We compared the fecal microbial profiles of urolithiasis patients, healthy controls, mice before and after gavage with urolithiasis patient stool, and mice before and after gavage with healthy control stool. By examining the synchronous changes in the abundance of microbial species before and after gavage, we identified 24 candidate species that may influence stone formation (Table 1).

After removing some species that have not yet been studied, we selected two species with the greatest change in abundance after fecal gavage, *Aslitipes indistincus* and *Odoribacter splanchnicus*.

*A*. *indistincus* is a Gram-negative bacterium that metabolizes glucose into succinic acid and acetic acid in PYG broth medium base. This bacterium is spherical or rod shaped, strictly anaerobic, and about 0.5-0.7 × 1.0-3.8 *μ*m in size. Gray, slightly opaque round colonies measuring 0.1-0.5 mm in diameter can be observed after four days of anaerobic culture in the modified GAM agar medium. The major end products of glucose fermentation by *A*. *indistincus* in the PYG broth medium base are succinic acid and acetic acid. *A*. *indistincus* is intolerant to 20% bile; does not hydrolyze heptaphylline or gelatin; does not reduce nitrate; does not produce indole, oxidase, or urease; and produces catalase. Furthermore, *A*. *indistincus* metabolizes cellobiose, glucose, lactose, maltose, D-mannose, melezitose, raffinose, 1-rhamnose, salicin, sucrose, trehalose, and D-xylose to synthesize organic acids [4].

*Odoribacter splanchnicus* is a Gram-negative, anaerobic bacterium of the Odoribacter genus. *O*. *splanchnicus* metabolizes various sugars, including glucose, galactose, arabinose, lactose, and mannose, producing metabolites such as acetic acid, propionic acid, succinic acid, butyric acid, isovaleric acid, and isobutyric acid. *O*. *splanchnicus* does not reduce nitrate and contains highly active enzymes involved in the pentose metabolism pathway. This bacterium is not sensitive to aminoglycosides and polymyxins but is sensitive to tetracycline, lincomycin, clindamycin, erythromycin, and rifampicin [5].

## 4. Discussion

The human body is inhabited by a vast number of microbes and the interaction between these microorganisms, and their host may be critical to the health and disease of the host. However, it was not until the emergence of new molecular techniques that the diversity of this microbiome began to gain the attention of researchers. A recent study demonstrated a complex bidirectional relationship between the gut microbiome and the host and reported that this relationship may be critical to human health and may be associated with the pathogenesis of disease. The gut microbiome is not only involved in food digestion and nutrient extraction but can also alter the host immune response, prevent infection, metabolize drugs, and participate and regulate metabolism of the host [6].

The article "The Relationship between Urinary Stones and Gut Microbiomeby 16S Sequencing" was retracted in 2024. Reasons: signs of a paper mill; suspected computer-generated content; unreliable results or conclusions; concerns about the data.

Studies demonstrated that kidney stones are mineral tuberculosis in the calyces and pelvis, which are found to be free or attached to the renal papilla. When urine is oversaturated with minerals, stones (called kidney stones or urinary stones) form in the urethra, causing crystals to form, grow, accumulate, and stay in the kidneys. Globally, approximately 80% of kidney stones are made of a mixture of calcium oxalate (CaOx) and calcium phosphate (CaP). Stones composed of uric acid, magnesium phosphate, and cystine are also common, accounting for about 9%, 10%, and 1% of the total number of stones, respectively. Stones may also be oversaturated with some relatively insoluble drugs or their metabolites, which may cause the urine components to crystallize in the renal collecting duct (iatrogenic stones) [7]. About 75% of kidney stones are mainly composed of calcium oxalate, and urinary oxalate is considered a risk factor.

According to the composition of stones, urinary stones are mainly divided into five categories: calcium oxalate, calcium phosphate, magnesium ammonium phosphate, uric acid, and cystine. Among them, oxalate occupies the vast majority, exceeding 85%. The microbiota refers to the entire microbial population that colonizes in a specific location and includes not only bacteria but also other microorganisms such as fungi, archaea, viruses, and protozoa [8]. The scientific community has shown great interest in the gut microbiota in recent years; the gut microbiota is associated with many human diseases, such as intestinal diseases such as inflammatory bowel disease (IBD) [9] and irritable bowel syndrome (IBS) [10], metabolic diseases such as obesity and diabetes [11], and allergic diseases [12] to neurodevelopmental diseases, although the strength of some evidence is not sound in many of them. It has long been believed that the gut microbiota has a significant functional role in maintaining the healthy intestines of normal individuals and humans as a whole. There is now more and more evidence that studies on humans and sterile mice support these speculations. The United States Human Microbiome Project (HMP) [13], European Human Gut Microbial Genomics (MetaHIT) [14], and several other studies have proven that normal intestinal flora is beneficial to health at the genetic level. These effects make it possible for the gut microbiota to also affect the absorption and secretion of solutes related to kidney stones.

The article "The Relationship between Urinary Stones and Gut Microbiomeby 16S Sequencing" was retracted in 2024. Reasons: signs of a paper mill; suspected computer-generated content; unreliable results or conclusions; concerns about the data.

To date, little is known about the general role of the gut microbiota in the pathophysiology of kidney stones. A recent study found that the gut microbiome of patients with kidney stones is significantly different from that of patients without stones. Whether these differences in bacterial abundance seen by stone formers and controls are the cause of stone formation or secondary to other variables such as antibiotic exposure or diet is uncertain. Allison and colleagues discovered the oxalobacteriumformigenes (Oxf) in 1985, which has attracted considerable attention due to its involvement in calcium oxalate stone disease. But for other bacteria that may affect the formation of urinary calculi, there are few reports.

In this study, we found that the gut microbiome of healthy controls and urolithiasis patients was significantly different and we determined the correlation between the gut microbiome and urolithiasis using fecal transplants in mice. A. indistinctus and O. splanchnicus are both Gram-negative anaerobes involved in food hydrolysis and metabolism in the intestine and may contribute to crystal formation in the kidneys. However, the factors influencing urolithiasis and the mechanisms by which these bacteria participate in metabolism need further investigation.

In summary, the urolithiasis patients in this study had a different gut microbiome when compared with that of healthy individuals. The altered microbiome increased the rate of crystal formation in renal tubules and accelerated urinary stone formation in the mouse model of urolithiasis.

## Figures and Tables

**Figure 1:** The Shannon index distribution among the experimental and control groups.

**Figure 2:** A comparison of the microbial composition at the phylum level between the experimental and control groups.

**Figure 3:** Rate of stone formation in each group.

**Figure 4:** Shannon index. (1) Healthy control stool. (2) Urolithiasis patient stool. (3) Mouse feces before PBS gavage. (4) Mouse feces after PBS gavage. (5) Mouse feces before urolithiasis patient stool gavage. (6) Mouse feces after urolithiasis patient stool gavage. (7) Mouse feces before healthy control stool gavage. (8) Mouse feces after healthy control stool gavage.

**Figure 5:** Phylum. (1) Healthy control stool. (2)Urolithiasis patient stool. (3) Mouse feces before PBS gavage. (4) Mouse feces after PBS gavage. (5) Mouse feces before urolithiasis patient stool gavage. (6) Mouse feces after urolithiasis patient stool gavage. (7) Mouse feces before healthy control stool gavage. (8) Mouse feces after healthy control stool gavage.

The article "The Relationship between Urinary Stones and Gut Microbiomeby 16S Sequencing" was retracted in 2024. Reasons: signs of a paper mill; suspected computer-generated content; unreliable results or conclusions; concerns about the data.

**Table 1:** Bacterial flora distribution.

Name of species	(1) Healthy control stool solution	(2) Urolithiasis patient stool solution	(3) 0 day after gavage with urolithiasis patient stool solution in mice	(4) 3 weeks after gavage with urolithiasis patient stool solution in mice	(5) 0 day after gavage with healthy control stool solution in mice	(6) 3 weeks after gavage with healthy control stool solution in mice	Total
Bacteroides_coprocola	538	0	1	0	0	0	539
Unidentified OUT 112	8	1	52	6	26	37	130
Uncultured bacterium OUT 148	1	0	45	25	14	17	102
OUT 215	1	0	24	1	10	24	60
Dorea formicigenerans	24	0	1	0	0	0	25
Unidentified OUT 416	1	0	1	0	2	2	6
Uncultured Bacteroidales bacterium	8	14	7930	8967	13373	5858	36150
Uncultured organism OUT 11	0	2	201	1304	1810	1601	4918
OUT 13	835	3166	0	1	1	1	4004
Uncultured bacterium OUT 32	0	1	217	228	430	69	945
Uncultured bacterium OUT 39	0	1	194	236	170	126	727
Uncultured bacterium OUT 46	0	3	303	517	147	134	1104
Firmicutes bacterium ASF 500	8	28	274	326	223	161	1020
Odoribacter splanchnicus	0	439	0	1	0	0	440
Gut metagenome	600	601	175	283	166	8	1833
(Clostridium) lactatifermentans	40	141	15	26	24	10	256
OUT 193	0	49	0	2	0	0	51
Oscillibacter ruminantium	0	1	2	41	22	9	75
Alistipes indistinctus	0	14	0	9	0	0	23
Uncultured bacterium OUT 359	1	7	0	2	0	0	10
Ruminococcaceae bacterium Marseille P2963	0	3	0	35	0	0	38
Uncultured bacterium OUT 432	0	8	0	2	0	0	10
Dorea sp. 5-2	0	2	264	396	48	50	862
OUT 128	33	1	46	35	28	26	218

## Data Availability

Our data would be available if checking process required.
